# CRP and ALT Levels in Individuals with Acute Biliary Pancreatitis after Endoscopic Retrograde Cholangiopancreatography and Endoscopic Sphincterotomy

**DOI:** 10.1155/2022/6492551

**Published:** 2022-06-11

**Authors:** Xiaofeng Zhu, Yuechen Sun

**Affiliations:** ^1^Department of General Surgery Division, Huzhou Central Hospital & Affiliated Central Hospital Huzhou University, Huzhou 313000, China; ^2^Department of Emergency Division, Huzhou Central Hospital & Affiliated Central Hospital Huzhou University, Huzhou 313000, China

## Abstract

**Objective:**

The goal of this study was to see how effective endoscopic retrograde cholangiopancreatography combined with endoscopic sphincterotomy was in treating acute biliary pancreatitis and how it affected CRP and ALT levels.

**Methods:**

This analysis is based on a 100-patient acute pancreatitis (ABP) study conducted at our institution from June 2019 to June 2020. They were divided into two groups of 50 cases each, the control group and the observational group, according to the random number table. Endoscopic sphincterotomy and ERCP were performed on the observation group instead of open surgery on the control group as a point of comparison (EST). The followings were compared including abdominal pain relief duration, blood amylase recovery duration, and hospital stay duration, as well as Serum C-reactive protein (CRP), interleukin-6 (IL-6), and tumor necrosis factor-*α* (TNF-*α*) level; the ALT, AST, and GGT levels of the two groups were compared, as well as the occurrence of problems in both groups.

**Results:**

The observation group had a significantly shorter duration of abdominal pain, blood amylase recovery, and hospital stay. Presurgery CRP, IL-6, and TNF-*α* levels in both groups were significantly lower in the observation group than in the control group. According to the results of the study, both groups saw significant decreases in ALT, AST, and GGT after surgery; however, the levels of these markers in both groups were significantly lower in the observation group after surgery than in the control group. The observation group's (14.00 percent) complication rate was substantially lower.

**Conclusion:**

ERCP and EST in the treatment of ABP can not only successfully improve clinical indexes and facilitate the recovery of patients but also reduce the levels of CRP and alt, reduce the level of inflammation, and enhance renal function, with reduced problems, which has a high clinical reference value.

## 1. Introduction

Acute biliary pancreatitis (ABP) is a common emergency in the department of gastroenterology, which is mainly caused by self-digestion of pancreatic tissue, pancreatic fluid overflow, impaired pancreatic mucosal barrier, and obstruction of pancreatic duct caused by inflammation and biliary calculi. The main clinical manifestations are jaundice, abdominal distension, and abdominal pain [1]. ABP can also cause bleeding and shock, which requires active and effective treatment; otherwise, it may lead to death [2]. The prevalence of ABP is steadily rising, posing a grave hazard to human life as a result of dietary and lifestyle changes [3]. Surgery is the most common treatment for ABP patients in clinical practice, with the goal of removing obstruction, ensuring proper drainage, and lowering bile duct pressure [4]. In the past, laparotomy was mostly adopted, which was characterized by significant curative effect, large surgical trauma, and slow recovery [5]. As medical technology continues to advance, minimally invasive treatment is becoming more and more common in clinical practice. Meanwhile, endoscopic retrograde cholangiopancreatography (ERCP) is a commonly used treatment at present, which can quickly remove the obstruction and effectively control the disease. Treatment for pancreatic bile duct disease is currently the “gold standard” [6, 7]. Meanwhile, endoscopic sphincterotomy (EST) can ensure the patency of pancreatic fluid. Compared with open laparotomy, it is less traumatic and results in a quicker recovery time after surgery [8]. The combination of ERCP and EST in ABP is still under investigation, but there are few data to support this approach. As a part of this study, CRP and ALT levels of patients will be evaluated to see how successfully ERCP and EST treatment of ABP affects their health outcomes. It provides a better basis for comparing the treatment of ABP.

## 2. Methods and Data

### 2.1. General Information

The 50 patients in the control group and the 50 patients in the observation group who were admitted from June 2019 to June 2021 were randomly assigned to two groups. The observation group underwent ERCP and EST in addition to standard open surgery in place of the control group. This study has the blessing of the hospital's ethics committee. A comparison of the two groups shows statistical indistinctness when it comes to gender, age, duration of illness before to admission, underlying cause, and degree of disease severity (Table 1).

### 2.2. Inclusion and Exclusion Criteria

Inclusion criteria are as follows: ① B-ultrasonography, CT, and MRI scans were used to diagnose all of the individuals with ABP; ② patients with normal organ functions, such as the heart, liver, and kidneys; and ③ patients or members of their families signed an informed consent form.

Exclusion criteria are as follows: ① participants in this study with medical conditions that prevent them from having surgery were excluded; ② patients with malignant tumor, blood system diseases, and immune system diseases; ③ ABP patients caused by systemic infection, hyperlipidemia, drugs, and alcohol addiction; and ④ pregnant or lactating women.

### 2.3. Methods

#### 2.3.1. Surgical Methods

All patients were given antibiotics, somatostatin, antispasmolysis, sedative, and so on. The patient's vital signs were closely monitored, and hematuria amylase, blood routine, and liver and kidney function tests were performed before surgery to ensure that the patient met the surgical indications.

The control group received traditional open surgery: patients were first given general anesthesia and then supine on the operating table. This procedure was completed by shearing off the upper portion of one's xiphoid process (0.8–1.5 cm) and securing the common bile duct with a fibrous catheter. The stone was removed with a stone basket and pulled out directly from the puncture sheath. After stone removal, routine examination of extrahepatic bile duct was performed to avoid residual stones. The tube was then inserted into the right abdominal wall from the Ventral foramen. The common bile duct was left with a 22 or 20 *T* tube. Aspirated through a puncture wound, one arm of the *T* tube extends from the right costal border (xiphoid process). Angiography was performed 4 weeks after surgery, and extubation was performed after normal conditions.

The observation group received ERCP combined with EST: anesthesia was administered first, and then the patients were positioned on the operating table. Retrograde cholangiopancreatography was performed by oral insertion of a duodenoscope and injection of 30% meglumine. After the size, number, hardness, location, and anatomical structure of the calculi were observed, the mastoid muscle was cut 10 ∼ 15 mm, and electric resection and electrocoagulation mixed current were adopted to perform net lithotomy under endoscopy. First, insert the balloon or stone basket for stone removal. For stones with a diameter of >1 cm, mechanical gravel basket can be used for stone removal. For the stones embedded in the ampulla, a needle-like knife can be used to precut the nipple and remove the stone. Then, according to the residual stones, whether to indurate the nasobiliary duct drainage can be decided.

Two groups of patients were given routine anti-infection therapy, nutritional support, fluid replenishment, and maintenance of acid-base and electrolyte balance.

#### 2.3.2. Detection Method

Blood was drawn from each patient and placed in an EP tube the morning before and the morning after surgery. For testing, serum was separated from blood samples and stored at −80 °C after standing for one hour at room temperature in an ultra-high-speed vm-1400-2kb centrifuge.

Inflammatory factors: CRP, interleukin-6, and enzyme-linked immumosorbent assay (ENZYme-Linked Immumosorbent assay) were regulated more effectively using an enzyme-linked immumosorbent assay (ELISA). A kit provided by Sophia Biotechnology Co. TNF- *α* and Il-6 were measured using LTD.

The AEROSET, an automated biochemical analyzer from Abbott in the United States, was used to measure ALT, AST, and GGT levels in the blood.

### 2.4. Observation Indicators

① Clinical indicators: between the two groups, researchers measured how quickly patients' abdomen pain subsided, as well as how quickly their blood amylase returned to normal. ② CRP, IL-6, and TNF-*α* levels were checked before and after the surgery in both groups. ③ Prior to and following surgery, the ALT, AST, and GGT levels in both groups were compared. (4) Complications: gastrointestinal bleeding, pancreatic abscess, biliary fistula, infection, and thoracoabdominal effusion were observed in both groups.

### 2.5. Statistical Methods

The statistical analysis was performed using SPSS 18.0. *T* was used to examine the significance of the data, which were shown as mean standard deviation (±*S*). As an example (*n*) or percentage (percent), enumeration data were evaluated by *χ*2. Significant differences were indicated by a *p* value of 0.05 or less.

## 3. Results

### 3.1. Comparison of Clinical Indicators

Table 2 shows that the observation group's time to pain alleviation, blood amylase recovery, and hospital stay were considerably shorter.

### 3.2. Comparison of Levels of Inflammatory Factors

Presurgery blood levels of CRP, IL-6, and TNF-*α* were not substantially different in the two groups (*P* > 0.05). After surgery, the levels of CRP, IL-6, and TNF- in both groups decreased. Serum CRP, IL-6, and TNF-*α* levels were significantly different between the observation and control groups (*P* < 0.05) as shown in Table 3 and Figure 1.

### 3.3. Comparison of Liver Function Indexes

Prior to surgery, ALT, AST, and GGT levels in the two groups were not significantly different. In both groups, post-surgery ALT, AST, and GGT levels dropped. Experiment group values of ALT, AST and GGT were found to be statistically considerably lower than those in the control group, as shown in Table 4 and Figure 2.

### 3.4. Comparison of Complications

When compared with the control group, the number of complications experienced by those in the observation group was considerably reduced (*P* < 0.05), as shown in Table 5.

## 4. Discussion

ABP is a chemical inflammation caused by obstruction of the biliary tract, which leads to the activation of trypsin in the acinar or pancreatic duct and the self-digestion of surrounding tissues. Early clinical manifestations may include minor symptoms such as stomach discomfort, nausea, and vomiting. Later clinical manifestations may include more severe symptoms such as shock, jaundice, and bleeding, as well as severe ABP [9]. Traditional surgical methods not only fail to cure ABP radically but also cause severe stress response due to major surgical trauma, which increases the risk of complications and death to a certain extent [10]. Since science and technology have advanced, minimally invasive techniques have been steadily introduced into clinical practice. ERCP and EST are minimally invasive procedures with less trauma, pain, and complications [11, 12]. Efficacy and effects on patient CRP and ALT levels of combined ABP treatment have been studied in a limited number of trials. This study found that ERCP and EST had a substantial impact on the treatment of ABP, as well as a significant impact on CRP and ALT levels at the same time. The following are the reasons for this.

Coutinho et al. [13] found that patients treated with ERCP had quicker pain alleviation and hospitalization times than those treated with conservative methods. Pancreatitis, gastrointestinal hemorrhage, and infection were reported to occur in approximately 16.0 percent of the children treated with endoscopic retrograde cholangiopancreatography (ERCP), extracorporeal shock therapy (EST), drainage, and lithotomy by Zeng et al. [14]. In this experiment, the observation group's hospital stay was shorter than the control group's, as was the time to alleviate stomach discomfort and normalize blood amylase levels. In the observation group, gastrointestinal hemorrhage, biliary fistula, infection, and effusions were less common. According to the evidence, ERCP and EST assist in curing ABP with fewer complications. Standard surgical procedure involves removing the gallbladder, separating and dissecting the common bile duct, and incising its front wall. This may be the explanation. After common bile duct incision, choledochoscope is used for exploration and stone extraction through the incision, which increases surgical trauma, causes bleeding, and increases the risk of postoperative complications [15]. In the case of pancreatic and biliary illnesses, ERCP has a high diagnostic efficiency since it can clearly exhibit lesions of the pancreas and bile duct, as well as the position and shape of calculi. In addition, the location, degree, and nature of the lesion can be observed, so as to effectively remove stones and facilitate rapid recovery of patients. EST can guarantee the patency of pancreatic fluid. ERCP combined with EST avoids the common bile duct incision and lowers iatrogenic harm when compared with standard surgery. In addition to these advantages, the operation is minimally invasive and has minor incision and trauma; a rapid postoperative recovery; and reduced postoperative complications [16, 17].

Inflammation, which is one of the most important components in ABP, can be caused by surgery, which is traumatizing to some extent, and this can lead to an increase in stress response and inflammation, which can lead to an increase in ABP symptoms [18]. TNF-*α* is one of the most prevalent clinical inflammatory factors, and the more TNF-*α* is present, the more strong the inflammatory response is [19]. Lowering CRP, IL-6, and TNF-*α* levels helps cure ABP clinically. CRP, IL-6, and TNF-*α* serum levels reduced following surgery for both groups. These data imply that the combination of ERCP and EST may successfully decrease the body's inflammation level, allowing for therapeutic treatment, despite the observation group's serum levels being lower than those of the control group. Analysis of the causes: ERCP combined with EST can effectively relieve biliary tract obstruction and make bile fully drained, which can promote the reduction of pancreatic duct pressure, thus effectively eliminating pancreatic duct drainage and promoting inflammation to subside [20].

Relevant studies have shown that the occurrence of ABP can easily cause liver damage, and pancreatic edema can lead to bile duct obstruction, resulting in obstruction of bile drainage and further damage to liver function [21]. ALT, AST, and GGT are common clinical liver function indicators, and the higher the level of ALT, AST and GGT, the more serious the liver function damage [22]. Bhutiani et al. [23] explored the therapeutic effect of ERCP + EST on patients with local pancreatic cancer undergoing irreversible electroporation. The study found significant improvement in liver function. The levels of ALT, AST, and GGT were lowered in both groups after surgery, and the observation group had lower levels than the control group, which was in accordance with the results of Bhutiani's research, suggesting that ERCP and EST may effectively boost the liver function of ABP. For this reason, patients can benefit from the removal of stones via ERCP and EST. At the same time, it also expands the application scope of minimally invasive surgery in biliary surgery and ensures normal physiological function of digestive tract and integrity of biliary tract. In addition, ERCP combined with EST, as a minimally invasive operation, has little trauma, can effectively reduce unnecessary injury, and avoid water, electrolyte, and physiological dysfunction caused by bile outflow [24, 25].

Because of the study's small sample size, there may be some disagreement between the data in the results and their true value. No long-term follow-up was conducted; hence, it was unable to determine ERCP's long-term efficacy in treating ABP. As a result, larger samples and longer follow-up periods are required for future validation investigations.

## 5. Conclusion

The combination of ERCP and EST has great efficacy in the treatment of ABP, which can successfully improve clinical indicators, lower CRP and ALT levels, and enhance liver function with fewer problems, which is worthy of reference in clinical circles.

## Figures and Tables

**Figure 1:** Comparison of inflammatory factor levels.

**Figure 2:** Comparison of liver function indexes.

**Table 1:** Comparing two sets of generic information.

General information		Control group	Observation group	*t*/*χ*^2^	*P*
Gender [*n* (%)]	Male	20 (40.00)	21 (42.00)	0.023	0.887
	Female	30 (60.00)	29 (58.00)		
Average age (years)		52.96 ± 7.47	53.22 ± 7.80	0.372	0.708
Mean time from onset to hospital admission (*h*)		27.32 ± 5.86	27.60 ± 5.57	0.459	0.639
Etiology [*N* (%)]	Simple cholecystolithiasis	26 (52.00)	24 (48.00)	0.473	0.492
	Common bile duct stone	14 (28.00)	16 (32.00)		
	Intrahepatic bile duct calculi	10 (20.00)	10 (20.00)		
Severity of disease [*N* (%)]	Light	34 (68.00)	32 (64.00)	0.454	0.501
	Heavy	16 (32.00)	18 (36.00)		

**Table 2:** Comparison of clinical indexes $\left(\bar{x}\pm s,d\right)$.

Clinical indicators	Control group	Observation group	*T*	*P*
Abdominal pain relief time	4.31 ± 0.53	2.47 ± 0.44	17.138	0.000
Time for blood amylase to return to normal	9.01 ± 1.10	5.46 ± 1.01	12.689	0.000
Length of hospital stay	16.97 ± 2.69	11.40 ± 2.41	16.031	0.000

**Table 3:** Comparison of inflammatory factor levels $\left(\bar{x}\pm s\right)$.

Indicators		Control group	Observation group
CRP (mg/L)	Before the operation	165.87 ± 23.64	166.08 ± 23.82
	After the operation	120.40 ± 20.53 ^*∗*#^	76.18 ± 11.59 ^*∗*#^
IL-6 (*μ*g/L)	Before the operation	13.78 ± 2.47	14.19 ± 2.51
	After the operation	10.47 ± 2.81 ^*∗*#^	5.73 ± 2.30 ^*∗*#^
TNF-*α* (*μ*g/L)	Before the operation	93.66 ± 10.44	93.86 ± 10.68
	After the operation	60.07 ± 7.73 ^*∗*^	21.64 ± 5.31 ^*∗*#^

**Table 4:** Comparison of liver function indexes $\left(\bar{x}\pm s,U/L\right)$

Indicators		Control group	Observation group
ALT	Before the operation	156.43 ± 21.69	157.17 ± 21.81
	After the operation	102.19 ± 18.90 ^*∗*#^	49.17 ± 6.32 ^*∗*#^
AST	Before the operation	58.31 ± 8.12	58.20 ± 8.18
	After the operation	46.43 ± 6.64 ^*∗*#^	37.50 ± 6.59 ^*∗*#^
GGT	Before the operation	58.41 ± 6.09	58.03 ± 6.05
	After the operation	50.22 ± 7.21 ^*∗*^	39.30 ± 5.63 ^*∗*#^

**Table 5:** Comparison of complications [*n* (%) ].

Complications	Control group	Observation group	*χ* ^2^	*P*
Gastrointestinal hemorrhage	2 (4.00)	1 (2.00)	—	—
Pancreatic abscess	4 (8.00)	1 (2.00)	—	—
Biliary fistula	3 (6.00)	1 (2.00)	—	—
Infection	3 (6.00)	0 (0.00)	—	—
Pleural and abdominal effusion	6 (12.00)	4 (8.00)	—	—
Total	18 (36.00)	7 (14.00)	6.542	0.014

## Data Availability

The data used to support the findings of this study are available from the corresponding author upon request.

## References

[1] Pirouz A., Sadeghian E., Jafari M. (2021). Investigating the factors affecting the development of biliary pancreatitis and their relationship with the type and severity of complications. *Middle East J Dig Dis*.

[2] Ruiz Rebollo M. L. (2022). Recurrent acute biliary pancreatitis - a frequent and preventable condition potentially associated with morbidity and mortality. *Revista Española de Enfermedades Digestivas*.

[3] Zver T., Calame P., Koch S., Aubry S., Vuitton L., Delabrousse E. (2022). Early prediction of acute biliary pancreatitis using clinical and abdominal CT features. *Radiology*.

[4] Lyu Y. X., Cheng Y. X., Wang B., Zhao S., Chen L. (2022). Safety of early same-admission laparoscopic cholecystectomy for acute mild biliary pancreatitis. A retrospective study for acute pancreatitis. *Videosurgery and Other Miniinvasive Techniques*.

[5] Nwuke C., Ibeh B. (2020). Antidiarrheal potential of methanol extract of combretum dolichopetalum and its fractions in wistar albino rats [J]. *SPR*.

[6] Emara M. H., Ali R. F., Mahmoud R., Mohamed S. Y. (2021). Postcholecystectomy biliary injuries: frequency, and role of early versus late endoscopic retrograde cholangiopancreatography. *European Journal of Gastroenterology and Hepatology*.

[7] Muangkaew P., Kamalaporn P., Mingphruedhi S. (2020). Outcomes of delayed endoscopic retrograde cholangiopancreatography in patients with acute biliary pancreatitis with cholangitis. *Asian Journal of Surgery*.

[8] Kucserik L. P., Marta K., Vincze A. (2019). Endoscopic sphincterotoMy for delayIng choLecystectomy in mild acute biliarY pancreatitis (EMILY study): protocol of a multicentre randomised clinical trial. *BMJ Open*.

[9] Fratantoni M. E., Giuffrida P., Di Menno J. (2021). Prevalence of persistent common bile duct stones in acute biliary pancreatitis remains stable within the first week of symptoms. *Journal of Gastrointestinal Surgery*.

[10] Ejaz H., Saharan Q. M., Ashiq S. (2021). Elimination of heavy metals and pesticides from wastewater by using Bagasse Fly Ash. *SPR*.

[11] Jin Z., Wei Y. P., Lin H. P. (2020). Endoscopic ultrasound‐guided versus endoscopic retrograde cholangiopancreatography‐guided biliary drainage for primary treatment of distal malignant biliary obstruction: a systematic review and meta‐analysis. *Digestive Endoscopy*.

[12] Khan M. A., Khan Z., Tombazzi C. R., Gadiparthi C., Lee W., Wilcox C. M. (2018). Role of cholecystectomy after endoscopic sphincterotomy in the management of choledocholithiasis in high-risk patients. *Journal of Clinical Gastroenterology*.

[13] Coutinho L. M. D A., Bernardo W. M., Rocha R. S. (2018). Early endoscopic retrograde cholangiopancreatography versus conservative treatment in patients with acute biliary pancreatitis. *Pancreas*.

[14] Zeng J. Q., Deng Z. H., Yang K. H. (2019). Endoscopic retrograde cholangiopancreatography in children with symptomatic pancreaticobiliary maljunction: a retrospective multicenter study. *World Journal of Gastroenterology*.

[15] Kabaria S., Mutneja H., Makar M. (2021). Timing of endoscopic retrograde cholangiopancreatography in acute biliary pancreatitis without cholangitis: a nationwide inpatient cohort study. *Annals of Gastroenterology*.

[16] Birda C. L., Sharma V. (2022). Urgent endoscopic retrograde cholangiopancreatography for acute biliary pancreatitis: few answers and more questions. *The National Medical Journal of India*.

[17] Ridtitid W., Kulpatcharapong S., Piyachaturawat P., Angsuwatcharakon P., Kongkam P., Rerknimitr R. (2019). The impact of empiric endoscopic biliary sphincterotomy on future gallstone-related complications in patients with non-severe acute biliary pancreatitis whose cholecystectomy was deferred or not performed. *Surgical Endoscopy*.

[18] Okamoto T., Fukuda K. (2021). Acute pancreatitis after biliary and pancreatic stent removal with a forward-viewing endoscope. *Case Rep Gastroenterol*.

[19] Sadeghian M., Sadeghi O., Esmaillzadeh A. (2019). Findings from the meta-analysis on whole-grain consumption and biomarkers of systemic inflammation are misleading. *Journal of the American College of Nutrition*.

[20] Zhou X. D., Chen Q. F., Zhang Y. Y. (2019). Outcomes of endoscopic sphincterotomy *vs* open choledochotomy for common bile duct stones. *World Journal of Gastroenterology*.

[21] Hashimoto S., Fujita T., Ido A. (2019). Emergent endoscopic ultrasonography-guided antegrade treatment for acute biliary pancreatitis in a patient with altered gastrointestinal anatomy. *Digestive Endoscopy*.

[22] Yuan X. F., Wen X., Ling Y. (2021). FXR mediated bile acid signal to advance the study of cirrhosis of the liver regeneration. *SPR*.

[23] Bhutiani N., Davidyuk V., Mortensen G. F. (2020). Safety, efficacy, and technical details of endoscopic retrograde cholangiopancreatography after irreversible electroporation for locally advanced pancreatic cancer. *Journal of Gastrointestinal Surgery*.

[24] Chandra S., Klair J. S., Soota K., Livorsi D., Johlin F. (2019). Endoscopic retrograde cholangio-pancreatography-obtained bile culture can guide antibiotic therapy in acute cholangitis. *Digestive Diseases*.

[25] Tringali A., Rota M., Rossi M., Hassan C., Adler D. G., Mutignani M. (2019). A cumulative meta-analysis of endoscopic papillary balloon dilation versus endoscopic sphincterotomy for removal of common bile duct stones. *Endoscopy*.

